The article "Effects of CT/MRI Image Fusion on Cerebrovascular Protection, Postoperative Complications, and Limb Functional Recovery in Patients with Anterior and Middle Skull Base Tumors: Based on a Retrospective Cohort Study" was published in 2022. Journal: Contrast Media Mol Imaging.

# Effects of CT/MRI Image Fusion on Cerebrovascular Protection, Postoperative Complications, and Limb Functional Recovery in Patients with Anterior and Middle Skull Base Tumors: Based on a Retrospective Cohort Study

**DOI:** 10.1155/2022/7855576

**Published:** 2022-09-13

**Authors:** Dandong Fang, Chen Yang, Haiyan Zhou, Xiaonan Liu, Jian Mao, Baosen Hou, Shimin Liu, Wei Huang

**Affiliations:** ^1^Department of Neurosurgery, The Sanmenxia Central Hospital, Sanmenxia 472000, Henan, China; ^2^Department of Neurosurgery Tangdu Hospital, The Fourth Military Medical University, Xi'an 710038, China; ^3^Department of Child Development and Behavior, The Sanmenxia Central Hospital, Sanmenxia 472000, Henan, China; ^4^The Minimally Invasive Neurosurgery Department of the 1st Affiliated Hospital of Kunming Medical University, Kunming 650032, Yunnan, China

## Abstract

**Objective:**

To explore the effect of CT/MRI image fusion on cerebrovascular protection, postoperative complications and limb function recovery in patients with anterior and middle skull base tumors.

**Methods:**

During January 2019 to December 2021, a retrospective study was conducted on 50 patients who underwent anterior and middle skull base tumor resection in the same surgeon group in our hospital. According to the different surgical approaches, the patients were assigned to the fusion group (*n* = 29) and the routine group (*n* = 21). The routine group was operated with traditional operation, and the fusion group was operated with CT/MRI image fusion technique. The operation time, wound volume, resection rate and Karnofsky performance status (KPS), blood transfusion (vascular protection), tumor resection rate, and postoperative complications were compared.

**Results:**

The time of operation in the fusion group was shorter compared to the routine group, and the volume of the wound cavity in the fusion group was smaller compared to the routine group, and the difference was statistically significant (*P* < 0.05). Following treatment, the KPS score of the fusion group was remarkably higher compared to the routine group, and the difference was statistically significant (*P* < 0.05). The intraoperative blood transfusion rate in the fusion group was 17.24%, and the intraoperative blood transfusion rate in the routine group was 47.62%, and the difference was statistically significant (*P* < 0.05). The resection rate in the fusion group (89.66%) was remarkably higher compared to the routine group (61.90%, *P* < 0.05). The incidence of postoperative complications in the fusion group (6.90%) was remarkably lower compared to the control group (33.33%, *P* < 0.05).

**Conclusion:**

The application of CT/MRI image-fusion technology can effectively enhance the clinical symptoms of patients with tumors in the anterior and middle region of the skull base, which can promote the prognosis, shorten the operation time, reduce unnecessary cerebral neurovascular injuries, and retain more brain functions.

## 1. Introduction

Resection of deep intracranial tumors, especially tumors in functional areas, is one of the unavoidable challenges in the growth of long-term brain surgeons, which requires long-term training to be competent [1]. The surgery is still the main therapeutic approach. The purpose of surgical treatment of intracerebral tumors is to remove the lesions as completely as possible while minimizing the loss of function and improving the life quality of patients after operation [2–4]. Because of the complexity of the brain tissue and the importance of its function, it is very important to accurately judge the location and boundary of the tumor and its relationship with the surrounding important nerves and vessels. The total resection rate of traditional surgery is low, and there are many postoperative complications. It is reported that the common complications are hemiplegia, aphasia, and even coma vegetative state [5–7]. How to remove intracranial tumors on the premise of preserving the patient's neurological function has become a major problem in neurosurgery. Tumors of the skull base are difficult to operate on because of their deep location, the uneven skull base, the abundance of blood vessels and nerves running through the skull base, and the narrow surgical space [8, 9]. Giant skull base tumors mostly destroy normal anatomical structures due to pushing and erosion of surrounding tissues [10]. However, how to determine the tumor approach before surgery has become a difficult problem.

Other medical imaging techniques are required during surgery for patients with mid-anterior skull base tumors. Medical imaging techniques help to improve the accuracy of diagnosis and maximize the efficacy of the procedure. At present, medical imaging models can be classified into two categories: anatomical imaging and functional images. Anatomical imaging shows the anatomical structure of the body, such as X-ray, computed tomography (CT), and magnetic resonance imaging (MRI). Additionally, functional imaging can provide metabolic information of tissues and organs, such as functional magnetic resonance imaging (FMRI) and diffusion tensor imaging (DTI). Anatomical imaging shows anatomical structures, but lacks the ability to show metabolic features of tissues and organs. Functional imaging can compensate for this, but functional imaging is not accurate enough for anatomical structures. In clinical work, the diagnosis and treatment of diseases must be combined with anatomy and functional imaging.

In order to comprehensively apply a variety of imaging modes to obtain more comprehensive image information, it is often necessary to integrate, compare, and analyze the effective information in clinical work. At first, image registration and lesion localization only by human brain analysis depend on the empirical judgment of the observer, so it is difficult to avoid errors in the understanding of tumor extent between observations and observers themselves [11]. In the 1990s, medical image fusion technology gradually appeared in people's line of sight. The so-called medical image fusion technology refers to the integration of a variety of anatomical and functional imaging data [12–15]. Image fusion largely depends on the development of computer image processing technology. Due to the differences in the development of computer technology, some medical image fusion technologies started early and developed relatively maturely. Some image processing technology lags and the related research starts late. Meanwhile, advanced medical image acquisition equipment is expensive and the fusion process is time-consuming and laborious, which restricts the development of medical image fusion technology to a great extent.

According to medical imaging equipment, fusion technology can be classified as homologous image fusion and heterologous image fusion [16, 17]. The new images obtained by fusion attach importance to disease diagnosis, treatment, and observation of curative effects [18]. In addition, the fusion of neuro-navigation can ensure the safety of the operation, maximize the protection of the patient's neurological function, and improve the patient's prognosis [19]. The purpose of this study was to compare the cerebrovascular protection, postoperative complications, and limb function recovery of patients undergoing skull base tumor resection with multimodal image fusion technology through a retrospective cohort study.

## 2. Patient and Methods

### 2.1. General Information

During January 2019 to December 2021, a retrospective study was conducted on 50 patients who underwent anterior and middle skull base tumor resection in the same surgeon group in our hospital. According to the different operative methods, the patients were assigned to the routine and the fusion group. The routine group was operated with traditional operation, and the fusion group was operated with CT/MRI image fusion technology—routine group (*n* = 21) and fusion group (*n* = 29). The ratio of male to female in the routine group was 6/15. The age ranged from 21 to 59 years with an average age of (43.38 ± 3.40) years. The location of tumor was anterior skull base (*n* = 17), middle skull base (*n* = 4), and tumor size ≤ 5 cm (*n* = 18) and > 5 cm (*n* = 3). In the fusion group, the ratio of male to female was 13/16. The age was 19 to 66 years, and the average age was 43.56 ± 3.59 years. The location of tumor was anterior skull base in 15 cases, middle skull base in 14 cases, and tumor size ≤ 5 cm in 22 cases and > 5 cm in 7 cases. There exhibited no significant difference in the basic data (*P* > 0.05).

### 2.2. Inclusion Criteria and Exclusion Criteria

Inclusion criteria include the following: 1) all cases must be diagnosed as skull base tumors by pathological biopsy; 2) selected cases had indications for radiotherapy (the tumor was located in the main functional area or next to important blood vessels and was sensitive to radiation); 3) the cases had agreed to undergo radiotherapy; 4) those who had the conditions to complete the CT-simulated localization scan and MRI scan; 5) the patients whose neck conditions were suitable for the C-type radiotherapy headrest; 6) all were primary, single, unilateral space-occupying lesions; and 7) no obvious surgical contraindications.

Exclusion criteria include the following :1) those who were allergic to contrast agents and could not complete enhanced CT localization scan or MRI scan; 2) those who had artifacts in the scan image data, which interfered with the judgment of the lesion; 3) those who had neurological dysfunction caused by other diseases in the past; and 4) those who had dysfunction of other vital organs.

### 2.3. Imaging Examination

All patients were scanned by CT and MRI one day before operation. During the examination, the supine position of the patients indicated the structures of scalp, skull, brain tissue, blood vessels, and tumors. The original DICOM data were recorded to an U disk or CD. The skull CT was performed with dual-source CT (256slice). The recording parameters were as follows: tube voltage, 120 kV; tube current, 425 mA; rotation time, 0.5 s/*r*; pitch, 0.969 0.5 s/*r*; scan field (FOV), 26 × 26 cm; slice thickness, S1mm; and uninterrupted continuous scanning, including the mandible downward and the parietal bone upward. The scanning parameters of MRI equipment are as follows: conventional T1-weighted imaging (T1W1)—repetition time/echo time (TR/TE) 600 ms/7 ms; T2-weighted imaging (T2W1)—repetition time/echo time (TR/TE) 6000 ms/98 m; slice thickness of 2 mm; continuous scanning, scanning time of about 5 min and scanning field (FOV) of 25 × 25 cm; enhancement: gradient echo sequence (GRE); TR/TE2000/3 ms; Fov25 × 25 cm; slice thickness of 2 mm; continuous scanning without interval; and scanning time of 15 min; and contrast agent, Gd-DTPA 0.2 ml/kg.

### 2.4. Image Fusion

The original DICOM data of CT and MRI one day before operation were imported into medical image processing software (GDslicer4.10.0) through U disk or CD for multimodal matching and 3D reconstruction. The steps included image registration and volume rendering reconstruction (Volume Rendering module) to generate 3D images, including facial skin, skull, brain tissue, blood vessels, nerves, and tumors. For key regions, image segmentation (Model Segmentation Maker module, Volume Clip with Model module), and image fusion (Add Scalar Volume module) were carried out to reproduce 3D stereoscopic images. In addition, DICOM reconstruction (Create a Dicom serious) was carried out if necessary.

### 2.5. Simulated Operation before Operation

Omni-directional and multi-angle observation was carried out on the reconstructed three-dimensional images, including facial skin, skull, brain tissue, nerves, blood vessels, and tumors, focusing on whether the skull base was damaged or not. The situation around the tumor was observed on the three-dimensional map of brain tissue, tumor, blood vessels, and nerves. Moreover, the plane tissue was displayed inward from the cortex under the determined head position. After arriving at the surgical area to understand the brain tissue and blood vessels around the tumor (hiding the tumor if necessary), the virtual operation was completed to achieve personalized accurate surgical design.

### 2.6. Neuro-Navigation

In the study group, 7 navigation markers were pasted near the projected scalp before enhanced MRI and the location was marked with Meilan injection. Before operation, the patients received intubation general anesthesia, positioned according to the specific location of the intracranial lesions and the head frame fixed the patient's head, so that the relative position between the patient and the operation bed remained unchanged. The neuro-navigation probe was used to touch the labeled site of Meilan injection to further proofread the intracranial lesions of the patients and the fusion images in the navigation system to form a one-to-one correspondence. The control group was treated with enhanced nuclear magnetic resonance scanning, routine intubation anesthesia, and head frame fixation as the study group.

### 2.7. Surgical Operation

According to the fusion images presented by navigation, the research group designed scalp incision and the best surgical approach, routine craniotomy. According to the location of the tumor shown by the navigation, draw the tumor surface projection and prepare for surgery. Search for tumors under the guidance of neuro-navigation with a variety of images. Resection of the lesion should be accompanied by avoidance of traction on surrounding tissues and structures. In addition, intraoperative application of dehydrating and intracranial hypotensive drugs such as mannitol and hypertonic saline should be avoided. During the operation, the navigation stick was used many times after craniotomy to verify the anatomical position and confirm the location of the tumor. According to the three-dimensional images of fiber conduction bundle and angiogenesis in navigation, the safe range of resection of skull base tumor was defined and the operation was strictly within the safe range. The control group adopted the traditional operation method as far as possible. The tumor resection was performed empirically according to the preoperative enhancement of MRI.

### 2.8. Observation Index

The main results are as follows: (1) the operation time and the volume of the wound cavity. The formula for calculating the volume of the wound cavity is the Tada formula: the longest diameter of the front and rear × the longest diameter of the left and right sides × the longest diameter of the upper and lower parts × *π*/6; (2) KPS score before and after operation [20]. The KPS score is an index to evaluate the life quality of patients with a full score of 100. If the score is less than 50, they need help from others. The score is 50–70 for semi-self-care and 71–100 for self-care; (3) intraoperative blood transfusion (cerebrovascular protection); (4) the tumor total resection rate was evaluated by the results of 3d MRI examination before and after operation. The tumor total resection rate = (number of tumor complete resection cases/total number of cases) × 100%.

In addition, the tissue around the surgical wound was tested. If no residual tumor cells were detected, it was regarded as complete resection. If there were residual tumor cells, it was considered to be a complete resection; (5) the postoperative complications were observed and recorded and followed up for 6 months.

### 2.9. Statistics

SPSS 23.0 statistical software was adopted to process the data. The measurement data were presented as (±*s*). The group design *t*-test was adopted for the comparison, and the analysis of variance was adopted for the comparison between multiple groups. The Dunnett test was adopted for comparison with the control group. The counting data were presented in the number of cases and the percentage, the *χ*2 test was adopted for comparison between groups, and the bilateral test was employed for all statistical tests.

## 3. Results

### 3.1. Comparison of Operation Time and Volume of Wound Cavity

In our experimental results, the operation time in the fusion group was 280.11 ± 16.82 min. While in the conventional operation group, the operation time was 385.47 ± 37.55 min. The operation time in the fusion group was less compared to the routine group, and the difference was statistically significant (*P* < 0.05). We found that the size of the wound cavity in the fusion surgery group was 15.33 ± 2.25 cm^3^. While in the conventional surgery group, we observed that the wound volume was 18.31 ± 4.02 cm^3^. The volume of wound cavity in the fusion group was smaller compared to the routine group, and the difference was statistically significant (*P* < 0.05) (see Table 1 for details).

### 3.2. KPS Score Comparison

The KPS scores in the fusion group were 85.22 ± 8.63 and 97.65 ± 3.42 pre- and post-treatments. The KPS scores of the patients in the routine group were 83.67 ± 10.58 and 90.31 ± 2.04 pre-and post-treatments. The postoperative KPS score of the fusion group was higher compared to the routine group, and the difference was statistically significant (*P* < 0.05). In addition, the KPS score before treatment in the fusion group was remarkably higher than that after treatment, and the difference was statistically significant (*P* < 0.05) (see Table 2 for details).

### 3.3. Comparison of Intraoperative Blood Transfusion

The study indicated that in the fusion group, 5 people received blood transfusion, 24 patients did not receive blood transfusion, and the blood transfusion rate was 17.24%. In the routine group, 10 people received blood transfusion, 11 did not receive blood transfusion, and the blood transfusion rate was 47.62%. The number of blood transfusions in the fusion group was remarkably lower compared to the routine group, and the difference was statistically significant (*P* < 0.05). It was suggested that the fusion technique had a significant protective effect on cerebral vessels in the operating area (see Table 3 for details).

### 3.4. Comparison of Resection Rate of Anterior and Middle Skull Base Tumors

The study indicated that in the fusion group, 26 patients underwent complete resection of skull base tumors, 3 patients underwent subresection, and the total resection rate was 89.66%. In the routine group, complete resection of skull base tumors was performed in 13 patients, subresection was 8, and total resection rate was 61.90%. The surgical resection rate in the fusion group was remarkably higher compared to the routine group, and the difference was statistically significant (*P* < 0.05) (see Figure 1 for details).

### 3.5. Comparison of Postoperative Complications

In the fusion group, postoperative complications were found in 2 cases, including dysphagia in 1 case, cerebrospinal fluid rhinorrhea in 1 case, and no complications in 27 cases; and the incidence of complications was 6.90%. There were 7 cases of postoperative complications in the routine group, including dysphagia in 2 cases, cerebrospinal fluid rhinorrhea in 2 cases, loss of taste in 1 case, abducent nerve or oculomotor nerve paralysis in 2 cases, and no complications in 14 cases; and the incidence of complications was 33.33%. The incidence of complications in the fusion group was remarkably lower compared to the routine group, and the difference was statistically significant (*P* < 0.05) (see Figure 2 for details).

## 4. Discussion

Central nervous system tumors can occur in the brain, meninges, spinal cord, and nerves, but most of them occur in the brain [1]. The disease has a huge negative impact on human health and life quality. In recent years, people pay more and more attention to physical examination and prolonged survival time with disease and the incidence and detection rate of skull base tumors are also on the rise. The treatment of the central nervous system includes surgery, radiotherapy, chemotherapy, and targeted therapy [21–23]. Formally based on the above thinking, this study integrated CT and MRI imaging technology to discuss and evaluate the application value of this fusion imaging technology in the surgical resection of skull base tumors. Skull base tumors are also one of the most difficult problems in neurosurgery because of their deep location, narrow operating space, and surrounding important nerve vessels [24–26]. Therefore, surgeons strive to ensure that the patient's neurovascular function is complete based on ensuring safe tumor resection.

It is well known that CT can display the bony structure and calcification of skull base tumors, while MRI can display soft tissue information more clearly [27]. It can not only evaluate the edema of the tumor and its surrounding brain tissue, nerve, and vascular compression, but also better evaluate the relationship between the focus and the dura mater. Preoperative MRA or CTA examination can understand the blood supply of the tumor and surrounding blood vessels [28–30]. On the images of fusion and three-dimensional reconstruction, we can observe not only the bone changes in the skull base, but also the blood supply artery of the tumor, the relationship between the tumor and the surrounding brain tissue, and the edema of the surrounding brain tissue. The virtual operation can be performed before operation, and the surgical approach can be designed. In addition, the images after multimodal image fusion can directly show the relationship among tumors, nerves, and blood vessels, the enlargement of foramen ovale, and the destruction of posterior clinoid process, and accurately show the outline of the tumor and its relationship with the surrounding tissue and the boundary of the tumor, the displacement of optic chiasma, and its relationship with the surrounding blood vessels. Through the fusion of the two, this study can perfectly combine the advantages of CT and MRI and help clinicians understand the relationship between tumor and surrounding tissue, blood vessels, and nerves. The huge tumor of the skull base is still a difficult problem for neurosurgeons today. It is difficult to separate not only because the skull base tumor often adheres closely to the surrounding important blood vessels, nerves, and important tissue structures, or because the narrow skull base space makes it difficult for the tumor to be exposed. This is also because most skull base tumors grow slowly. The vital structures adjacent to the tumor become slender or even pushed into linear structures due to prolonged compression. A slight carelessness in the operation can lead to injury [10]. For large skull base tumors, total resection cannot be pursued blindly, when the arachnoid interface of the tumor adheres closely to the brainstem. The tumor invades the cranial nerve or internal carotid artery and the tumor invades the vein, sigmoid sinus, and transverse sinus. The residual part of the tumor is a wise choice [31–33]. In this study, the huge skull base tumor in the fusion group can identify the tissue, blood vessels, and nerves around the tumor after preoperative multimodal image fusion and maximize the resection of the tumor under the guidance of neuro-navigation. Compared with the surgical resection in the routine group, the fusion group can track the surgical process in real time, ensure the safety of the operation, and maximize the removal of the tumor at the same time to ensure the safety of patients.

Through the dynamic guidance of intraoperative real-time fusion imaging technology, fusion imaging can locate the tumor more accurately and display the adjacent tumor in real time, which shortens the time for the operator to think about the location, scope, and adjacent structure of the tumor during the operation [34]. It reduces unnecessary brain tissue damage caused by exploration and search for tumors to speed up the postoperative recovery of the patients. This study is suggested that the fusion technique has a significant protective effect on cerebral vessels in the operating area. The volume of the wound cavity is not the only criterion for judging the quality of surgery, but accurate and minimally invasive surgery is the direction of every surgeon. At present, there are few reports about the tumor cavity volume. This study showed that there exhibited no statistical difference in the preoperative tumor volume between the fusion imaging group and the routine group, but there is a significant difference in the postoperative tumor cavity volume. It is mainly due to the fact that the CT and MRI fusion imaging navigation system can locate the tumor accurately during the operation, dynamically display the adjacent relationship of the tumor, guide the operation in real time, achieve the maximum safe range of tumor resection, and reduce the damage to normal brain tissue. The fusion imaging navigation system shows obvious advantages in reducing the volume of the wound cavity.

The complications of craniocerebral surgery refer to the injury, loss, and dysfunction of other tissues and organs caused by the operation [35]. Postoperative intracranial infection and neurological impairment are obvious postoperative complications in neurosurgery [36, 37]. This study indicated that the complications in the fusion imaging group were lower compared to the routine operation group and there exhibited a statistically significant difference. The analysis showed that the main factors of infection might be that the operation takes a long time to find the tumor. When the wound cavity became larger, some patients with more bleeding even need blood transfusion. The incidence of postoperative neurological impairment in the fusion imaging group was lower compared to the conventional operation. The intracranial tumor was cut under the guidance of the neuro-navigation system, resulting in smaller brain tissue and nerve injury [38]. In this study, intracranial infection occurred mainly in the early stage of technical application in the fusion imaging group, but there was no obvious regularity in the traditional group. Due to the lack of proficiency in operation, the operation time is longer, the exposure time of the operation area is prolonged and the risk of infection is increased. With the development of new technology, the proficiency of navigation technology, and the strengthening of aseptic consciousness, the postoperative intracranial infection rate will be effectively enhanced. However, the number of cases enrolled in this study is still small with the progress of follow-up research.

The number of cases is relatively small, which cannot better reflect the superiority of neuro-navigation in terms of tumor total resection rate. The function of neuro-navigation is to “escort” the safety of the whole operation, while for highly difficult skull base tumors, especially huge skull base tumors, we cannot deny the important role of navigation according to the fact that the tumor is not completely removed. In this study, the total resection rate of tumor in the routine group has been at a high level, while the total resection rate in the fusion group is higher, which has reflected the importance of navigation. Our study still has some shortcomings. Firstly, the quality of this study is limited due to the small sample size we included in the study. Secondly, this research is a single-center study and our findings are subject to some degree of bias. Therefore, our results may differ from those of large-scale multicenter studies from other academic institutes. Our research is still clinically significant and further in-depth investigations will be carried out in the future.

Conclusively, the application of CT/MRI image fusion technology can effectively enhance the clinical symptoms of patients with tumors in the anterior and middle region of the skull base, which can promote the prognosis, shorten the operation time, reduce unnecessary cerebral neurovascular injuries, and retain more brain functions [39].

## Figures and Tables

**Figure 1:** Comparison of surgical resection rate between two groups of patients.

**Figure 2:** Incidence of complications in two groups of patients.

**Table 1:** Operation time and trauma cavity volume.

Group	*N*	Operation time (min)	Volume of wound cavity (cm^3^)
Fusion group	29	280.11 ± 16.82	15.33 ± 2.25
Regular group	21	385.47 ± 37.55	18.31 ± 4.02
*t*	—	13.404	3.341
*P*	—	＜0.01	＜0.01

**Table 2:** KPS scores between the two groups.

Group	N	KPS Score (points)		*t*	*P*
		Before treatment	After treatment		
Fusion group	29	65.22 ± 8.63	77.65 ± 3.42	7.210	＜0.01
Regular group	21	63.67 ± 8.58	70.31 ± 2.04	3.450	＜0.01
*t*		0.628	8.757		
*P*		>0.05	＜0.01		

**Table 3:** Comparison of intraoperative blood transfusion.

	*N*	blood transfusion	No blood transfusion	Blood transfusion rate
Fusion group	29	5	24	17.24%
Regular group	21	10	11	47.62%
*χ* ^2^	—	—	—	5.352
*P*	—	—	—	＜0.01

## Data Availability

The datasets used and analyzed during the current study can be obtained from the corresponding author upon reasonable request.
